# Interferon-Induced Transmembrane Protein 3 Expression Upregulation Is Involved in Progression of Hepatocellular Carcinoma

**DOI:** 10.1155/2021/5612138

**Published:** 2021-03-16

**Authors:** Yuli Hou, Shanshan Wang, Mengdan Gao, Jing Chang, Jianping Sun, Ling Qin, Ang Li, Fudong Lv, Jinli Lou, Yonghong Zhang, Yan Zhao

**Affiliations:** ^1^Department of Clinical Laboratory, Beijing You'an Hospital, Capital Medical University, Beijing 100069, China; ^2^Department of Clinical Laboratory, Xuanwu Hospital, Capital Medical University, Beijing 100053, China; ^3^Beijing Institute of Hepatology, Beijing You'an Hospital, Capital Medical University, Beijing 100069, China; ^4^Department of Pathology, Beijing You'an Hospital, Capital Medical University, Beijing 100069, China; ^5^Biological Information Center, Beijing You'an Hospital, Capital Medical University, Beijing 100069, China

## Abstract

**Purpose:**

Interferon-induced transmembrane protein 3 (IFITM3) is a key signaling molecule regulating cell growth in some tumors, but its function and mechanism in hepatocellular carcinoma (HCC) remain unknown. Our study investigated the relationship between the expression of IFITM3 and HCC development. *Material and Methods*. IFITM3 expression was identified via multiple gene expression databases and investigated in HCC tissue samples. Then, PLC/PRF/5 cells were transfected with lentivirus to knock down and overexpress the expression of IFITM3. IFITM3 expression, cell proliferation, and migration were detected by qRT-PCR, western blotting, QuantiGene Plex 2.0 assay, immunohistochemistry, CCK-8, and wound healing tests. RNA-seq technology identified the PI3K/AKT/mTOR pathway as an IFITM3-related signaling pathway for investigation.

**Results:**

IFITM3 expression was higher in HCC tissues than in adjacent normal tissues, and the level of IFITM3 was higher in HCC tissues with low differentiation and metastatic potential than in those with high/medium differentiation and without metastatic potential. A higher RNA level of IFITM3 was found in samples with IFITM3 rs12252-CC genotype rather than the TT genotype. Knockdown of IFITM3 in PLC/PRF/5 cells inhibited cell proliferation and migration, blocked the expression of the PI3K/AKT/mTOR signaling pathway, and decreased the expression of vimentin. The results were opposite with the overexpression of IFITM3.

**Conclusion:**

Upregulation of IFITM3 plays a role in the development of HCC. Possibly through regulating HCC cell proliferation and migration, these effects are associated with the PI3K/AKT/mTOR signaling pathway. Upregulation of IFITM3 is also associated with the IFITM3 rs12252-CC genotype.

## 1. Introduction

Hepatocellular carcinoma (HCC) is the second leading cause of cancer-related death according to World Health Organization (WHO) data [1, 2]. The occurrence and development of HCC are the result of all kinds of factors, among which genes and their polymorphisms play an important role in the susceptibility and progression of hepatic cancer [3]. Interferon-induced transmembrane protein 3 (IFITM3), a 10-15 kDa protein, is a double transmembrane protein that belongs to the IFITM family [4, 5]. It is now understood that IFITM3 exerts a significant role in a variety of cellular processes, from cell adhesion, homing and maturation of germ-cells, and immune-cell regulation to bone mineralization [6, 7]. Recently, increasing studies have reported that IFITM3 is abnormally expressed in various types of human cancers [8–10] and that it participates in tumor development. Metastasis is the most common reason for death in patients with HCC who have undergone curative resection [11–13]. The epithelial-mesenchymal transition (EMT) is likely to be induced by the regulation of signaling pathways through oncogenes leading to tumor progression and metastasis [14]. The expression of vimentin which is upregulated in EMT is an EMT marker [15].

The IFITM3 polymorphism rs12252-C encodes an isoform that is missing 21 amino acids from the amino terminus [16], which causes IFITM3 to function differently from the wild type. The rs12252-CC genotype has also been associated with low differentiation and progression of HCC [17].

Based on these previous studies, it is likely that IFITM3 has an important role in HCC progression and that its polymorphisms may have different effects. Therefore, this study is aimed at exploring the mechanism between IFITM3 and the development of HCC.

## 2. Material and Methods

### 2.1. HCCDB Database Analysis

HCCDB is a database of HCC expression chartbook containing 15 open HCC gene expression datasets containing complete 3917 samples, counting the information from the Quality Expression Omnibus (GEO), Liver Hepatocellular Carcinoma Venture of The Cancer Genome Chartbook (TCGA-LIHC) and Liver Cancer-RIKEN, and JP Venture from Universal Cancer Genome Consortium (ICGC LIRI-JP). HCCDB gives the visualization from a few computational investigations.

### 2.2. UALCAN Database Analysis

UALCAN (http://ualcan.path.uab.edu) uses TCGA level 3 RNA-seq and clinical data from 31 cancer types, allowing analysis of relative expression of genes across tumor and normal samples, as well as in various tumor subgroups based on individual cancer stages, tumor grade, or other clinicopathological features.

### 2.3. Hepatic Tissue Specimens

Thirty-eight HCC tissue specimens and fourteen HCC tissue specimens with adjacent noncancer tissues were surgically obtained between October 2017 and October 2018 at the Beijing You'an Hospital, Capital Medical University (Beijing, China). The samples were from eligible patients who met the diagnostic criteria of HCC based on the European Association for the Study of the Liver (EASL) guidelines. Patients were excluded if they had other cancers or a history of chemotherapy/radiotherapy for other cancers. The corresponding normal hepatic tissue samples were extracted >5 cm from the edge of the tumor, and no evident organization of the tumor cells was detected. The differentiation degree was defined by pathologists. All patients were diagnosed with hepatitis B virus infection. But considering the research that suggests interferon can impact the expression of IFITM3, all patients were recruited without the use of interferon (Table 1).

### 2.4. Quantitative Reverse Transcription Polymerase Chain Reaction (qRT-PCR)

Total RNA was isolated from the specimens with TRIZOL reagent (15596026, Thermo Fisher) and then reverse transcribed (AT301-03, TransGen Biotech). qRT-PCR was performed using the SYBR (QPK-201, TOYOBO) on an ABI V7 machine. Quantification was calculated by 2^-*ΔΔ*CT^ to indicate relative expression levels, by subtracting the CT value of the control gene from the CT value of IFITM3. The primer sequences for PCR amplification of IFITM3 gene and GAPDH are listed in Table 2. Total RNA was isolated from the specimens with TRIZOL reagent (15596026, Thermo Fisher) and then reverse transcribed (AT301-03, TransGen Biotech). qRT-PCR was performed using the SYBR (QPK-201, TOYOBO) on an ABI V7 machine. Quantification was calculated by 2-*ΔΔ*CT to indicate relative expression levels, by subtracting the CT value of the control gene from the CT value of IFITM3. The primer sequences for PCR amplification of the IFITM3 gene and GAPDH are listed in Table 2.

### 2.5. Western Blotting

Briefly, total cellular proteins were extracted using RIPA assay buffer containing protease inhibitors. Identical quantities of proteins were separated by SDS-PAGE electrophoresis and transferred onto nitrocellulose filter membranes. After incubation with antibodies specific for IFITM3, vimentin, PI3K, AKT, mTOR, p-PI3K, p-AKT, p-mTOR (all from CST, USA), and GAPDH (Sigma, USA), the blots were incubated with horseradish peroxidase- (HRP-) conjugated goat anti-rabbit (or mouse) IgG and then were detected by chemiluminescence. All primary and second antibodies for western blotting are listed in Table 2.

### 2.6. Cell Lines and Cell Culture

The HCC cell line PLC/PRF/5, HepG2 cell line, and QGY-7701 cell line were kindly provided by Dr. Gang Li (Department of Biochemistry and Molecular Biology, Peking University). All the cell lines were maintained in DMEM medium supplemented with 10% FBS in a 5% CO_2_ incubator.

### 2.7. Cell Counting Kit-8 (CCK-8) Assay

Cell Counting Kit (CCK)-8 (CK04, Dojindo) was used to assess the effect of IFITM3 on cell proliferation. Cells were seeded in a 96-well plate at 5 × 10^3^ cells/well with 100 *μ*l of complete culture medium. The cells adhered for 24 h, then 10 *μ*l CCK-8 was added to each well, and this was incubated at 37°C for 2 h. The 450 nm absorbance of each well was measured with a microplate reader. Each condition was performed in triplicate, and the experiments were repeated three times.

### 2.8. Wound Healing Test

Cell migration was evaluated using the wound healing test. Plant cells into 12-well microplates up to 80% confluence before scratch. Cell images were captured under a light microscope at 0, 24, 48, and 72 h following treatment.

### 2.9. Lentivirus Construction and Infection

Modified LV-IFITM3 vector lentiviral constructs (Beijing SyngenTech Co., LTD, Beijing, China) were used to knockdown IFITM3 in PLC/PRF/5 cells. The pLenti-CMV-IFITM3 vector lentiviral constructs to overexpress IFITM3. The virus was added to the cells for 24 h; then, this was replaced with a fresh culture medium. The cells were selected for stable transfection with 4 *μ*g/ml blastmycin over 2 weeks.

### 2.10. Immunohistochemistry

The HCC tissue samples were fixed in 10% formalin solution and embedded in paraffin. 0.3% hydrogen peroxide in methanol was used to block endogenous peroxidase for 20 min at room temperature. Antigen retrieval was performed in citrate buffer (pH 6.0) and heated with a microwave for 10 min. 4°C incubation was carried out overnight to bind primary antibodies (IFITM3, 1 : 400, CST, USA). The secondary anti-rabbit antibody (1 : 1,000) was then applied for 30 min at room temperature. The slides were rinsed with TBST, then treated with a solution of diaminobenzidine and counterstained with hematoxylin. The intensity of immunostaining was analyzed by the Servicebio Company who provided integrated optical density (IOD) values for evaluation.

### 2.11. QuantiGene Plex 2.0 Assay

The QuantiGene Plex 2.0 assay (Panomics/Affymetrix, Fremont, CA, USA) was used to confirm the microarray analysis. The assay was performed according to the manufacturer's instructions, accessible at https://tools.thermofisher.com/content/sfs/manuals/QuantiGene_Plex_User_manual.pdf. Briefly, tissue-extracted RNAs were added to a 96-well plate along with QuantiGene hybridization solution. The sealed hybridization plate was shaken at 54°C, 600 rpm overnight (18-22 h). The hybridization mixture was transferred to a prewetted filter plate, filtered, and washed three times in wash buffer. The samples were then incubated in three successive working solutions. Beads were identified, and fluorescent signals were measured. The raw data file contained signal intensity and background level for each gene in each sample.

### 2.12. RNA Sequencing

Six samples [three samples infected with LV-NC as the control group and three samples infected with LV-IFITM3 vector lentiviral as an experimental group] of PLC/PRF/5 were sequenced at BGI (Beijing Genomics Institute, Shenzhen, Guangdong, China) using standard RNA-seq technology. The NOISeq method was adopted to screen the differentially expressed genes (DEGs) between the LV-IFITM3 and LV-NC samples. Gene ontology (GO) annotation analysis was performed for the screened DEGs. Pathway classification and enrichment analysis of DEGs were performed based on the Kyoto Encyclopedia of Genes and Genomes (KEGG) database. DEGs were selected with the criteria of a fold-change of ≥2 and a *q* value (%) of <5% by statistical analysis.

### 2.13. Statistical Analysis

Analyses were performed with the Graph Pad Prism version 5 (Graph Pad Software, La Jolla, California, USA). Tailed Student's *t* test, chi-square test, and Fisher's exact test were used to analyze in experimental groups. A two-tailed value of *P* < 0.05 was considered to indicate a statistically significant result.

### 2.14. Ethics, Consent, and Permissions

The study was approved by the Beijing You'an Hospital Research Ethics Committee (Beijing, China). All the participants provided written informed consent. The methods were carried out following the approved guidelines and regulations. Consents to publish data in the form of documents and images were obtained from the participants or legal representatives.

## 3. Results

### 3.1. IFITM3 Was Overexpressed in Hepatic Tissues of HCC Patients and Was Survival-Associated

We initially evaluated IFITM3 transcription levels in multiple HCC studies from TCGA. Analysis in the HCCDB database revealed that mRNA expression of IFITM3 was significantly higher in HCC tissues than in adjacent normal tissues (Figures 1(a) and 1(b)). Data in the Oncomine database indicated that levels of IFITM3 DNA copy number were significantly higher in tumor tissues than in normal tissues (Figure 1(c)). Further subgroup analysis of multiple clinic-pathological features of TCGA-LIHC samples in the UALCAN database consistently showed elevated transcription levels of IFITM3. The expression of IFITM3 was significantly higher in HCC patients than in normal controls in subgroup analysis based on gender, age, weight, tumor grade, and TP53 mutation (Figure 1(d)). In order to verify the expression level of IFITM3 protein in HCC samples and nontumor samples, we examined the expression of IFITM3 protein in 14 pairs of hepatic tissues compared with adjacent normal hepatic tissues. IFITM3 was positively stained in the HCC tissues but weakly stained in the adjacent normal tissues (Figures 1(e) and 1(f)). Quantification suggested the IFITM3 IOD value was higher in HCC tissues than in adjacent hepatic tissues (*P* = 0.003, Figure 1(g)). The RNA level of IFITM3 was markedly upregulated in cancer tissues compared with corresponding noncancer adjacent hepatic tissues (*P* = 0.038, Figure 1(h)). IFITM3 protein expression was higher in cancer tissues in comparison with adjacent normal hepatic tissues (Figure 1(i)). Then, Kaplan-Meier survival curves were used to assess the association between IFITM3 expression and the survival outcomes of HCC cohorts with survival information available (Figure 1(j)). Generally, the high IFITM3 expression group had significantly shorter overall survival (*P* < 0.05) compared to the low expression group in the LIHC cohort.

### 3.2. IFITM3 Positively Regulates HCC Cell Migration and Proliferation

The protein expression of IFITM3 in the QGY-7701, HepG2, and PLC/PRF/5 human HCC cell lines was analyzed by western blotting analysis, and the expression level of IFITM3 protein was higher in PLC/PRF/5 cell line, so the PLC/PRF/5 cell was selected as the optimal experimental cell (Figure 2(a)). We infected IFITM3 shRNA and pLenti-CMV-IFITM3 into PLC/PRF/5 cell and found that the level of IFITM3 expression in the LV-IFITM3 was significantly lower than that in normal PLC/PRF/5 cell (*P* < 0.05, Figures 2(b)–2(d)). Additionally, the expression of IFITM3 was higher in pLenti-CMV-IFITM3 cells than in normal PLC/PRF/5 cells (*P* < 0.05, Figures 2(b)–2(d)). To demonstrate the involvement of IFITM3 in the migration of hepatic cells, a wound healing test was performed. The wound healing test showed that compared with normal cells, IFITM3 knockdown significantly inhibited HCC cell migration and the overexpression of IFITM3 could significantly promote the cell migration (*P* < 0.001, Figures 2(e) and 2(f)). Furthermore, cell proliferation was inhibited with IFITM3 knockdown and the overexpression of IFITM3 could promote the cell proliferation ability (*P* < 0.001, Figure 2(g)). These results suggested that IFITM3 could positively regulate the cell migration and proliferation ability in HCC cells.

### 3.3. RNA Sequencing and the Verification with qRT-PCR

The above results indicate that the knockdown of IFITM3 can inhibit the proliferation and migration of HCC cells. Therefore, we decided to screen for DEGs between the LV-NC and the LV-IFITM3 cells using NOISeq. The volcano plot of all expressed genes based on the results of each pair is shown in Figure 3(a). A total of 891 significantly upregulated genes and 3998 downregulated genes compared with the LV-NC were screened under the criteria of a minimum 2-fold-change and a *P* value < 0.001. Based on the GO-biological process (BP), cellular component (CC), and molecular function (MF), we found that among the DEGs with known BP classes, the largest group (624 genes) contained genes involved in cellular processes (Figure 3(b)). As genes usually interact with each other to perform their biological functions, we performed pathway classification and enrichment analysis of DEGs based on the KEGG database (Figure 3(c)). We selected pathways relating to cell motility, transport and catabolism, cell growth and death, and cancer overview to do KEGG enrichment and found that the PI3K-AKT signaling pathway played an essential role in regulating the EMT of HCC progression with a large number of DEGs (9 genes) (Figure 3(d)). Real-time PCR verification was undertaken of genes related to the PI3K/AKT signaling pathway including PI3K, AKT, and mTOR. We found that the RNA level of PI3K was downregulated (*P* < 0.01), the expression of AKT was also downregulated but not to a significant level (*P* > 0.05), and the expression of mTOR was downregulated (*P* < 0.01) with the knockdown of IFITM3 (Figure 3(e)).

### 3.4. Effects of IFITM3 on PI3K/AKT/mTOR Signaling and Vimentin Expression

We subsequently further investigated whether the function of IFITM3 in HCC cells was associated with the activation of PI3K/AKT/mTOR signaling by western blotting using ly294002, a new molecular inhibitor [18], to block PI3K/AKT/mTOR signaling at a concentration of 10 *μ*mol/l for 48 h. Vimentin is an EMT marker; its expression markedly decreased together with PI3K/AKT/mTOR with the use of ly294002 to block PI3K/AKT/mTOR signaling (Figures 4(a) and 4(c)). Additionally, the activity of PI3K/AKT/mTOR signaling was downregulated with the knockdown of IFITM3 and upregulated with the overexpression of IFITM3 compared with the untreated control (Figures 4(b) and 4(d)). Furthermore, the altered expression of IFITM3 was also related to the expression of vimentin.

### 3.5. IFITM3 rs12252-CC Genotype Was Associated with the Upregulation of IFITM3

The previous study has shown that the IFITM3 rs12252-CC genotype is associated with the progression of HCC [17]. To investigate the association between IFITM3 rs12252-CC genotype and the expression of IFITM3 in our samples, we examined the expression of IFITM3 RNA by QG-Plex and it was found that the expression of IFITM3 RNA increased with the degree of pathological differentiation of HCC (*P* = 0.038, Figure 5(a)). Furthermore, the level of IFITM3 was upregulated in HCC tissues with metastasis compared to those without metastasis (*P* = 0.005, Figure 5(b)). A significant upregulation of IFITM3 expression was observed in the IFITM3-CC genotype, as compared with the IFITM3-TT genotype (*P* = 0.043, Figure 5(c)). These results support the view that the IFITM3-CC genotype can influence HCC development and suggest this may be through increasing the expression of IFITM3.

## 4. Discussion

The analysis of databases and tissue samples from patients with HCC confirmed that IFITM3 mRNA levels are significantly higher in HCC than in normal liver tissue. Besides, high expression of IFITM3 was significantly related to poor survival in multiple cohorts. Furthermore, the high expression of IFITM3 was associated with the differentiation and metastasis of HCC. The results of this study support the previous studies that have shown IFITM3 is overexpressed in HCC and the overexpression of IFITM3 is significantly correlated with tumor metastasis and proliferation in HCC [17, 19, 20]. Furthermore, higher IFITM3 expression was found in IFITM3 with the rs12252-CC genotype rather than the TT genotype as shown in a previous study [17]. These findings suggest that the IFITM3 rs12252-CC genotype can upregulate the IFITM3 expression to participate in the development of HCC.

RNA sequencing showed that the PI3K/AKT/mTOR pathway was associated with the knockdown of IFITM3. The PI3K/AKT/mTOR axis can be activated by several intracellular signaling pathways. This activation is important for the regulation of several cellular events, including the cell cycle, proliferation and growth, and the EMT of malignant tumors [21–23]. There was less expression of vimentin when the PI3K/AKT/mTOR pathway was inhibited by ly294002, which illustrates that the PI3K/AKT/mTOR pathway plays an important role in EMT. Furthermore, the activity of PI3K/AKT/mTOR signaling and the level of vimentin were decreased with the knockdown of IFITM3, and there are opposite results with the overexpression of IFITM3, which suggests IFITM3 participates in the regulation of EMT. We hypothesize from the results that the relationship between IFITM3 and PI3K/AKT/mTOR signaling pathway is as shown in Figure 4(e). However, what drives IFITM3 expression in HCC and how its loss affects the PI3K/ATK signaling pathway remain unclear.

In conclusion, the present study investigated the role of the IFITM3 gene in the pathogenesis of HCC. The expression of IFITM3 appears to promote tumor progression in HCC. This may be through increased proliferation and migration of HCC cells via the PI3K/AKT/mTOR pathway. In addition, an increased expression of IFITM3 was observed in HCC tissues with the rs12252-CC genotype. These findings provide new and important information on the progression of HCC and suggest that IFITM3, particularly rs12252-CC genotype, may be beneficial as a novel molecular target for the treatment and diagnosis of HCC patients.

## Figures and Tables

**Figure 1:** IFITM3 was overexpressed in hepatic tissues of HCC patients and was survival-associated. (a, b) Chart and plot showing the expression of IFITM3 in tumor tissues and the adjacent normal tissues in HCCDB. (c) Box plot showing IFITM3 mRNA levels in the Roessler Liver 2. (d) IFITM3 transcription in subgroups of patients with HCC (UALCAN). Immunohistochemical results of IFITM3 expression were detected in HCC tissues (e) and adjacent normal tissues (f); magnification: ×100 (*n* = 14). (g) IFITM3 IOD level was tested in HCC tissues and adjacent normal tissues using IPP6.0 (*n* = 28). IFITM3 expression levels were assessed in tumor tissues and adjacent normal hepatic tissues using qRT-PCR (h) and western blotting (i) (*n* = 28). (j) IFITM3 is associated with survival outcome in TCGA LIHC cohort.

**Figure 2:** IFITM3 positively regulates HCC cell proliferation and migration. (a) IFITM3 expression was evaluated by western blotting analysis in three HCC cell lines. (b–d) Examination of IFITM3 expression in stably transfected HCC cells using western blotting and qRT-PCR. ^∗^*P* < 0.05, ^∗∗^*P* < 0.01, and ^∗∗∗^*P* < 0.001. (e, f) Wound healing tests were performed to detect cell migration in LV-IFITM3 and pLenti-CMV-IFITM3 HCC cells. Magnification, ×40. (g) CCK-8 assays were used to monitor cell proliferation in indicated cells. ^∗∗∗^*P* < 0.001 vs. normal. The data were analyzed using Student's *t* test, and the data are shown as the mean ± SEM, with three independent experiments in each group.

**Figure 3:** RNA sequencing and the verification of the qRT-PCR results. (a) Volcano plots of all expressed genes in each pairwise. (b) GO functional classification on the DEGs. (c) KEGG classification for cellular processes. (d) KEGG enrichment of cell motility, transport and catabolism, cell growth, and death and cancer overview. (e) qRT-PCR verification of the genes related with PI3K/AKT signaling pathway including PI3K, AKT, and mTOR. ^∗^*P* < 0.05 vs. LV-NC. The data were analyzed using Student's *t* test, and the data are shown as the mean ± SEM, with three independent experiments in each group.

**Figure 4:** Effects of IFITM3 on PI3K/AKT/mTOR signaling and vimentin expression. (a, c) Western blotting detection for the effect of ly294002 on PI3K/AKT/mTOR expression and vimentin. (b, d) Western blotting for the effects of IFITM3 on the expression of PI3K/AKT/mTOR signaling-related proteins in LV-IFITM3 and pLenti-CMV-IFITM3 cells. (e) Crosstalk between IFITM3, PI3K/AKT/mTOR signaling pathway and vimentin protein in HCC cells. ^ns^*P* > 0.05, ^∗^*P* < 0.05, ^∗∗^*P* < 0.01, and ^∗∗∗^*P* < 0.001 vs. normal. The data were analyzed using Student's *t* test, and the data are shown as the mean ± SEM, with three independent experiments in each group.

**Figure 5:** IFITM3 rs12252-CC genotype was associated with HCC progression. (a) Analysis of IFITM3 expression in HCC tissues of different differentiation grades using QG-Plex (*n* = 38). (b) The expression of IFITM3 was detected in HCC tissues with metastasis and without metastasis using QG-Plex (*n* = 38). (c) The IFITM3 RNA level was analyzed in rs12252-CC and TT genotypes using QG-Plex (*n* = 18).

**Table 1:** Antibodies and sequences used for western blotting, qRT-PCR, and shRNA for LV-IFITM3 and control LV-NC.

Protein		Mfrs./made in	Cat no.
*Primary antibodies*			
p-PI3K		Cell Signaling Technology/USA	4228P
P-AKT		Cell Signaling Technology/USA	4060P
p-mTOR		Cell Signaling Technology/USA	5536P
PI3K		Cell Signaling Technology/USA	4255
AKT		Cell Signaling Technology/USA	9272
mTOR		Cell Signaling Technology/USA	2972
GAPDH		Sigma/USA	G9545
Vimentin		Cell Signaling Technology/USA	5741S
IFITM3		Cell Signaling Technology/USA	59212S
Second antibodies			
HRP-conjugated anti-mouse IgG		Zhongshan Boil Tech Co./China	IH-0031
HRP-conjugated anti-rabbit IgG		Zhongshan Boil Tech Co./China	IH-0011
*Gene*		*Primer sequences*	
*RT-qPCR*			
IFITM3	Forward	5′-AGATGGTTGGCGACGTGAC-3′	
	Reverse	5′-AGGCCTGGAAGATCAGCACT-3′	
GAPDH	Forward	5′-TGAAGGTCGGAGTCAACGGA-3′	
	Reverse	5′-CCTGGAAGATGGTGATGGGAT-3′	
AKT	Forward	5′-TGTGGACCAACGTGAGGCTC-3′	
	Reverse	5′-AGGCAGCGGATGATGAAGGT-3′	
PI3K	Forward	5′-GGAAGCAGCAACCGAAACAA-3′	
	Reverse	5′-AGAGCAGGCATAGCAGCCCT-3′	
mTOR	Forward	5′-GCATCAGGACCTCTTCTCCT-3′	
	Reverse	5′-GCCCGACTGTAACTCTCTCC-3′	
shRNA			
LV-IFITM3		5′-GTGCTGATCTTCCAGGCCTA-3′	
LV-NC		5′-CCTCGTTCACCGCCGTCGCG-3′	

**Table 2:** Characteristics of the hepatocellular carcinoma (HCC) patients.

	All HCC patients (*n* = 52)
Mean age (years ± SD)	52.62 ± 9.3
Sex	
Female, *n* (%)	11 (21.2%)
Male, *n* (%)	41 (78.8%)
ALT (U/L, 25%-75%)	40.35 (24.03-54.08)
AST (U/L, 25%-75%)	38.10 (27.73-55.43)
TBIL (*μ*mol/L, 25%-75%)	20.05 (12.35-26.93)
DBIL (*μ*mol/L, 25%-75%)	3.70 (2.33-8.43)
AFP (ng/ml, 25%-75%)	20.72 (3.35-285.95)
Distal metastasis, *n* (%)	8 (15.4%)
Differentiation	
High, *n* (%)	26 (50%)
Medium, *n* (%)	17 (32.7%)
Low, *n* (%)	9 (17.3%)

ALT: alanine transaminase; AST: aspartate transaminase; TBIL: total serum bilirubin; DBIL: direct serum bilirubin; AFP: alpha-fetoprotein.

## Data Availability

The data used to support the findings of this study are available from the corresponding author upon request.
